# Effect of Integrated Nursing Care Based on Medical Alliance Mode on the Prevention and Treatment of Complications and Self-Efficacy of Patients with Coronary Heart Disease after PCI

**DOI:** 10.1155/2022/7727953

**Published:** 2022-03-09

**Authors:** Yujie Zhao, Xiaonan Wang

**Affiliations:** ^1^Department of Imaging Nursing, Jiaozhou Central Hospital of Qingdao, Qingdao City 266300, Shandong Province, China; ^2^Department of Geriatrics, The Second Affiliated Hospital of Mudanjiang Medical College, Mudanjiang City 157010, Heilongjiang Province, China

## Abstract

**Objective:**

To explore the effect of integrated nursing care based on the medical alliance model on prevention and treatment of complications and self-efficacy in patients with coronary heart disease (CHD) after PCI.

**Methods:**

The data of CHD patients treated in our hospital from January 2019 to January 2021 were analyzed in this retrospective study. One hundred and twenty patients were selected as the research subjects according to the inclusion and exclusion criteria and equally split into the observation group and reference group according to the order of admission. Both groups received routine nursing care, while the observation group was additionally given integrated nursing care based on the medical alliance model to compare the self-efficacy scores, scores of self-management abilities, and incidence of postoperative complications between the two groups before and after nursing. Both groups were nursed for 6 months.

**Results:**

Compared with the reference group, the observation group after nursing achieved a notably higher GSES score (26.10 ± 1.30 vs 22.18 ± 1.30, *t* = 16.516, *P* < 0.001), higher scores of self-management ability (*P* < 0.001) , and a lower incidence of postoperative complications (*P* < 0.05).

**Conclusion:**

Integrated nursing care based on the medical alliance model can improve the self-efficacy of CHD patients undergoing PCI, enhance their self-management ability, and reduce the incidence of postoperative complications, which is conducive to improving the prognosis of patients.

## 1. Introduction

Coronary heart disease (CHD), an ischemic heart disease, is caused by coronary atherosclerosis. Patients have different degrees of lumen occlusion and stenosis, resulting in myocardial ischemia, hypoxia, and necrosis, with the main clinical manifestations as chest pain (paroxysmal colic or crush pain) and chest distress [1]. According to China's fifth health service survey in 2013, the number of CHD patients over 15 years old in China exceeded 10 million [2], and China's Health and Family Planning Statistical Yearbook (2016) confirmed that the number was still on the rise. In the same period, the mortality of CHD patients in urban and rural areas in China also showed an increasing trend, with annual deaths of over one million, ranking second in the world [3]. At present, PCI is an important measure to reduce the mortality of CHD patients because it can effectively dredge the narrow and occluded coronary artery lumen and achieve myocardial perfusion [4, 5]. Shajrawi Abedalmajeed et al. have reported that PCI reduces the mortality of patients with acute myocardial infarction from 30.0% to 5.0%, but it cannot completely reverse coronary atherosclerosis, and the surgical operation damages the vascular wall of patients, resulting in various vascular complications after surgery and affecting the prognosis [6]. Postoperative secondary defense is the key to reducing postoperative complications in patients. For example, smoking cessation, alcohol restriction, and a healthy diet are effective behaviors to prevent the recurrence of adverse cardiovascular events after surgery. However, CHD patients often have negative emotions such as anxiety, and poor self-efficacy. Jiang Ying et al. have found that the self-management ability and nursing compliance of such patients decrease with the passage of time after discharge [7, 8]. Therefore, strong external intervention measures are required.

Since most CHD patients in China return to their homes and to the community for further rehabilitation after PCI, community nursing should improve the self-efficacy of patients through external intervention, which plays an important role in follow-up home care [9]. However, due to inadequate development of community rehabilitation in China and uneven knowledge and skills of community nursing staff, many CHD patients treated with PCI fail to receive consistent, effective, and high-quality nursing measures. In recent years, as the reform of public hospitals progresses, the medical alliance has provided more possibilities for community nursing [10], aiming to extend the way of nursing management in tertiary hospitals within the medical alliance to the community so as to improve the nursing quality of nurses in basic hospitals and meet the nursing needs of current practice. Based on the medical alliance, the nursing practice in our hospital can be homogenized to community nursing, so that CHD patients can obtain continuous medical care services at different medical locations and maintain good self-efficacy after receiving external nursing intervention. At present, the medical alliance model has been applied to the nursing of some CHD patients. Based on the model, the integrated nursing management of doctors and nurses can construct the trinity working pattern of doctors, nurses, and patients, and maximize the advantages of this clinical nursing. Based on this, this paper will explore the effect of integrated nursing care based on the medical alliance model on the prevention and treatment of complications and self-efficacy of CHD patients after PCI.

## 2. Materials and Methods

### 2.1. Research Design

This retrospective study was conducted in our hospital from January 2019 to January 2021, trying to explore the effect of integrated nursing care based on the medical alliance model on the prevention and treatment of complications and self-efficacy in CHD patients after PCI.

### 2.2. General Data

The data of 120 CHD patients treated from January 2019 to January 2021 were retrospectively analyzed. All patients meeting the following inclusion criteria were included: (1) patients meeting the diagnostic criteria for CHD formulated by the World Health Organization (WHO) [11], and undergoing PCI treatment to reconstruct blood circulation; (2) patients with no postoperative heartache; (3) patient with the stable condition and good mental state; (4) patients with normal limb function; and (5) patients with complete clinical data. Exclusion criteria: (1) patients who could not communicate with others due to hearing impairment, language disorders, unclear awareness, and other factors; (2) patient dropping out midway or falling off during follow-up; (3) patients with upper limb swelling and skin infection before surgery; (4) patients with severe organ dysfunction; and (5) patients with severe complications before surgery. According to the order of admission, 120 patients were equally split into the observation group and reference group. The observation group included 32 males and 28 females with an average age of 65.55 ± 5.26 years old and an average disease course of 3.68 ± 1.24 years, including 12 cases at the education level of junior high school, 28 cases of senior high school (including secondary technical school), and 20 cases of junior college or above. There were 42 cases of acute myocardial infarction and 18 cases of unstable angina pectoris. 28 cases had diseased vessels in the anterior descending artery, 3 cases in the circumflex artery, 9 cases in the right coronary artery, and 20 cases in multiple arteries. The reference group included 30 males and 30 females with an average age of 66.15 ± 5.22 years old and an average disease course of 3.60 ± 1.70 years, including 10 cases at the education level of junior high school, 29 cases of senior high school (including secondary technical school), and 21 cases of junior college or above. There were 40 cases of acute myocardial infarction and 20 cases of unstable angina pectoris. 26 cases had diseased vessels in the anterior descending artery, 5 cases in the circumflex artery, 10 cases in the right coronary artery, and 19 cases in multiple arteries.

### 2.3. Moral Considerations

This study followed the Declaration of Helsinki [12], and patients signed the informed consent.

### 2.4. Exit Criteria

Judged by the research team, patients with the following conditions were unsuitable to continuously participate in the experiment, and their medical records would be kept but not for data analysis: (1) the patients had suddenly deteriorated condition during the experiment; (2) some severe complications or complications occurred; and (3) the subjects proposed to withdraw from the clinical trial to the research group.

### 2.5. Methods

#### 2.5.1. Reference Group

Routine nursing was performed in the reference group, namely, general nursing intervention during the perioperative period of PCI for CHD patients. The patients received a routine examination before surgery and health education on the precautions of PCI to alleviate their fear. During surgery, the patients' physical sign data were closely monitored, and the appropriate temperature and humidity of the operating room were ensured to prevent their body temperature from decreasing. After surgery, the limb pain, swelling, and extravasation of the wound dressing in the patients were observed, and the patients were informed to pay attention to bed rest, especially the operative limb needing more than 6 h to move. The nursing staff used the pressure hemostatic device to decompress regularly, observed whether the patient had a forearm hematoma, and removed the hemostatic device at 24 h after surgery. Pain relief measures were taken for the patients with pain in accordance with the doctor's advice, while psychological nursing was adopted to relieve their anxiety and restlessness.

#### 2.5.2. Observation Group

This group received routine nursing care combined with integrated nursing care based on the medical alliance model. (1) A team of integrated nursing care based on the medical alliance model was established (hereinafter referred to as the team). The team consisted of cardiologists, cardiac surgeons, and nursing staff from the hospital, nutritionists, psychological consultants, and community physicians and nurses, with all team members of bachelor's degree or above. A WeChat group was established on the day of determining personnel to facilitate real-time communication. (2) *Team training.* Before nursing, all members received training from the therapists to learn the application of finger exercises and ultrasonic physiotherapy apparatus. The nursing staff received training from cardiologists, cardiac surgeons, nutritionists, and psychological consultants. The teaching content was formulated based on the *Chinese Expert Consensus on Coronary Heart Disease Rehabilitation and Secondary Prevention*, which mainly included the theoretical knowledge of PCI treatment for CHD, postoperative pain management requirements, medication management requirements, dietary requirements, and precautions for preventing complications. The assessment was carried out after training, and the qualified nurses could nurse the patients. (3) *Intervention during hospitalization.* ① the electronic files were immediately established on the day of enrollment to record the general information, psychological status, and nutritional status of patients, among which the psychological status was determined based on the scores of the *Hamilton anxiety* and *depression scales.* ② During medication of patients, the staff paid close attention to their adverse reactions after using drugs such as vasodilators, including dizziness and low blood pressure, to improve the prevention awareness of adverse reactions. ③ Since CHD patients suffer from a heavy psychological burden, the staff should listen to them enthusiastically and actively, and provide individualized psychological guidance according to their knowledge level to alleviate their negative emotions, maintain mental stability, and create good conditions for treatment. ④ The diseases such as hypertension and hyperlipidemia, the predisposing factors of CHD, were closely related to the daily living habits of patients. Therefore, nurses needed to develop a healthy diet for them, guide them to carry out a low-salt and low-fat diet, and maintain appropriate exercise to reduce the risk factors. ⑤ On the first day after surgery, the medical and nursing staff jointly viewed the patients, and the doctors explained the surgery and the causes of postoperative limb pain to them and gave them the decomposed diagram of the finger exercises. ⑥ To reduce the risk of postoperative complications in CHD patients, the nurses used plain words to educate patients and their families to improve their cognitive level of CHD, enhance their ability to monitor the disease and actively identify the risk factors for complications, and improve the quality of family care. ⑦ After surgery, the heart rate and ECG of the patients were closely observed, and drugs such as atropine were prepared before extubation. During extubation, atropine was given immediately if symptoms such as decreased heart rate and blood pressure, pale face, and sweating occurred. (4) *Community services.* ① The nursing department of our hospital provided the guidance on nursing training, nursing techniques, nursing quality management, and other aspects for community nursing staff, and then transferred the patients' information to the community service centers on the day of discharge. The community nursing staff visited the patients once a week to understand their recovery and nutrition, and they recorded their condition in the follow-up file. ② During the follow-up, the staff evaluated the patients' disease and living conditions, advised them to keep the room clean and tidy, investigated whether they had complications, and checked their rehabilitation diary. ③ After the nutritionists evaluated the nutritional status of patients, the nursing staff formulated reasonable diet plans to improve their tolerance. ④ The nursing staff communicated with patients and provided psychological counseling for those with negative psychology to enable them to actively face life after PCI and improve their compliance with rehabilitation treatment. ⑤ Community lectures were conducted every 2 months to provide health education for the patients by team members. After the lectures, the patients were encouraged to communicate with each other and learn from positive cases to improve medication compliance.

### 2.6. Observation Criteria

#### 2.6.1. Self-Efficacy Scores

*General self-efficacy scale (GSES)* [13] was applied to evaluate the self-efficacy of both groups before and after nursing, with the internal consistency coefficient as CronbachA = 0.87, which contained 10 problems related to self-efficacy. The Likert's four-level scoring method was used, with a score range of 1 (completely wrong) to 4 (completely correct). The total score was 40 points, and a higher score demonstrated stronger general self-efficacy.

#### 2.6.2. Score of Self-Management Ability

The self-management ability of both groups before and after nursing was evaluated using the *coronary heart disease self-management scale (CSMS)* [14], with an internal consistency coefficient as CronbachA = 0.91, which included seven dimensions and 27 items. The Likert's five-level scoring method was used, and a higher score demonstrated stronger self-management ability. The seven dimensions of CSMS were the management of bad habits (20 points), daily life management (20 points), symptom management (20 points), disease knowledge management (25 points), emergency management (15 points), nursing compliance management (15 points), and emotional cognitive management (20 points).

#### 2.6.3. Incidence of Postoperative Complications

The types of postoperative complications were recorded to calculate the incidence of complications.

### 2.7. Statistical Processing

In this study, the data were processed by software SPSS 20.0, and graphed by GraphPad Prism 7 (GraphPad Software, San Diego, USA). The data included in the study were the enumeration data and measurement data, tested by *X*^*2*^ and *t*-test. When *P* < 0.05, the differences were statistically significant.

## 3. Results

### 3.1. Patient Self-Efficacy Scores

With no statistical difference in the GSES scores before nursing between the two groups (20.10 ± 1.21 vs 19.92 ± 1.35, *t* = 0.769, *P* = 0.443), the GSES score of the observation group was notably higher compared with the reference group (26.10 ± 1.30 vs 22.18 ± 1.30, *t* = 16.516, *P* < 0.001) after nursing.

### 3.2. Self-Management Ability Scores

Figure 1 shows higher scores of self-management abilities in the observation group after nursing (*P* < 0.001).

No obvious differences were observed in the scores of management of bad habits, daily life management, symptom management, disease knowledge management, emergency management, nursing compliance management, and emotional cognitive management between the observation and reference groups before nursing (14.12 ± 1.21 vs 13.98 ± 1.36, 13.02 ± 1.27 vs 12.88 ± 1.14, 10.02 ± 1.26 vs 9.85 ± 1.30, 16.22 ± 1.28 vs 16.05 ± 1.19, 7.08 ± 1.23 vs 7.00 ± 1.20, 8.17 ± 1.20 vs 7.90 ± 1.06, 14.25 ± 1.27 vs 14.13 ± 1.28, *P* > 0.05).

The scores of the seven dimensions in the observation group after nursing were notably higher compared with the reference group (18.00 ± 1.22 vs 14.82 ± 1.26, 17.02 ± 1.32 vs 14.82 ± 1.30, 16.15 ± 1.31 vs 13.70 ± 1.82, 22.87 ± 1.23 vs 18.68 ± 1.43, 13.05 ± 1.18 vs 10.10 ± 1.23, 13.20 ± 1.27 vs 10.28 ± 1.63, 18.18 ± 1.15 vs 15.62 ± 1.43, *P* < 0.001).

### 3.3. Incidence of Postoperative Complications

The observation group had a lower incidence of postoperative complications compared with the reference group (*P* < 0.05), as shown in Table 1.

## 4. Discussion

Though PCI is an effective measure to alleviate coronary artery stenosis, it cannot completely reverse the situation of coronary artery stenosis and occlusion, with the incidence of restenosis in patients as 20.0%–60.0% at one year after surgery [15]. Therefore, postoperative prevention is necessary to reduce the frequency of adverse cardiovascular events and other complications. Postoperative prevention mainly depends on the clinical guidance of doctors and nurses, but patients still play a main role in their daily management. Their self-management behaviors are influenced by many factors. For example, a negative psychological state can reduce the self-efficacy of patients and gradually erode their belief in treatment [16, 17], while a low cognitive level may mislead patients into believing that PCI is a radical cure for CHD and restores their original living habits, which is not conducive to maintaining their nursing compliance [18]. Since CHD is a chronic disease, patients still need to maintain a positive attitude towards prevention and treatment after PCI. However, routine nursing is often unable to achieve this purpose. Scholars Jokanovic Natali et al. believe that in routine nursing, the nursing staff focus on basic nursing and education is often inconsistent with the doctors' health education due to a lack of communication, affecting the patients' public confidence in health education and compliance with clinical nursing [19]. Integrated nursing care can put doctors, nursing staff, and patients in the same working pattern. Nursing staff can fully participate in the process of disease treatment and enhance the effectiveness of nursing intervention, while doctors can join in the management of patients to better understand their rehabilitation, with better effect. Bosselmann Lena et al. have confirmed that the integrated nursing care model can improve the self-management ability of patients, enhance their trust in nursing staff, and facilitate the effect of health education [20]. This study showed a higher self-efficacy score in the observation group (*P* < 0.001) because the patients in this group had a better ability to accept health education under integrated nursing care, thus effectively alleviating their negative emotions such as anxiety, doubt, and depression. Therefore, the patients' negative emotions were reduced, and their self-efficacy was improved.

In recent years, the promotion of medical alliances provides a better basis for the development of doctor-nurse integration, which enables doctors and nursing staff of public hospitals to help community doctors and nurses. The excellent brand effect enables patients to trust the community staff and receive the integrated nursing measures with the same quality during hospitalization as after discharge, which is conducive to forming a long-term and coherent nursing mode [21, 22]. The *13th Five-Year Nursing Development Plan* proposes to improve the contents and methods of nursing services with specialist nurses as the carrier and provide community residents with preventive knowledge on common diseases and early rehabilitation of chronic diseases and home care services so as to enhance the nursing compliance of patients with chronic diseases after discharge [23]. Siow Elaine et al. have found that high-quality community care can assist in screening risk cases and intervene with patients at different levels to implement scientific nursing management [24]. Targeted community nursing is more likely to benefit CHD patients because most patients can still maintain a high level of health knowledge during hospitalization after surgery, while enhancing their self-management ability on the basis of external intervention, thereby reducing the incidence of postoperative complications. This study found that the observation group after nursing achieved a notably higher self-efficacy score (*P* < 0.001) and a lower incidence of postoperative complications (11.7%, *P* < 0.05), which was consistent with the findings of Yu Mingming et al. Yu Mingming et al. believe that self-management ability is the main cause of cardiovascular adverse events after surgery, with an obvious negative correlation between them [25]. The high-quality and long-term nursing mode can enhance the self-efficacy of patients by reducing their negative emotions and improving their health knowledge level. At the same time, their nursing compliance is maintained by external intervention to keep high self-management ability and improve the prognosis of patients.

## 5. Conclusion

In conclusion, integrated nursing care based on the medical alliance model provides more possibilities for the integration of medical care, and this medical reform is conducive to improving the long-term nursing effects of CHD patients. It can improve the self-efficacy of CHD patients undergoing PCI, enhance their self-management ability, and reduce the incidence of postoperative complications, which is conducive to improving the prognosis of patients.

## Figures and Tables

**Figure 1:** Scores of self-management ability ($\overset{–}{x}$ ± *s*, points). *Note.* Figure 1(a), management of bad habits; Figure 1(b), daily life management; Figure 1(c), symptom management; Figure 1(d), disease knowledge management; Figure 1(e), emergency management; Figure 1(f), nursing compliance management; and Figure 1(g), emotional cognitive management.

**Table 1:** Incidence of postoperative complications [n(%)].

Items	Observation group (*n* = 60)	Reference group (*n* = 60)	X^2^	*P*
Subcutaneous congestion	3(5.0)	5(8.3)	0.536	0.464
Local hematoma	1(1.7)	2(3.3)	0.342	0.559
Venous embolism of upper limb	0(0.0)	2(3.3)	2.034	0.154
Vascular occlusion	0(0.0)	2(3.3)	2.034	0.154
Arrhythmia	1(1.7)	3(5.0)	1.035	0.309
Vascular vagus reflex	1(1.7)	2(3.3)	0.342	0.559
Contrast-induced nephropathy	0(0.0)	1(1.7)	1.008	0.315
Heart failure	1(1.7)	2(3.3)	0.342	0.559
Total incidence	7(11.7)	19(31.7)	7.070	0.008

## Data Availability

Data to support the findings of this study are available on reasonable request from the corresponding author.
